The article "Evaluation of an Experimental Gel Containing Euclea natalensis: An In Vitro Study" was published in 2012. Journal: Evid Based Complement Alternat Med.

# Evaluation of an Experimental Gel Containing *Euclea natalensis*: An *In Vitro* Study

**DOI:** 10.1155/2012/184346

**Published:** 2012-11-05

**Authors:** Sílvia Helena de Carvalho Sales-Peres, Letícia Ferreira de Freitas Brianezzi, Juliane Avansini Marsicano, Moacir Rossi Forim, Maria Fatima das Graças Fernandes da Silva, Arsenio Sales-Peres

**Affiliations:** ^1^Department of Pediatric Dentistry, Orthodontics and Public Health, Bauru School of Dentistry, University of São Paulo, Al. Octávio Pinheiro Brisolla, 17012-901 Bauru, SP, Brazil; ^2^Department of Chemistry, Laboratory of Natural Products, Federal University of São Carlos, Rodovia Washington Luiz, 13565-905 São Carlos, SP, Brazil

## Abstract

*Objective*. To evaluate the effect of an experimental gel containing *Euclea natalensis* extract on dentin permeability. *Methods*. Thirty-six dentin discs, 1-mm-thick. The discs were prepared from the coronal dentin of extracted human third molars that were divided into 3 groups (*n* = 10). The dentin discs in each group were treated with the groups following experimental materials: (FG): 1.23% fluoride gel, pH 4.1; (EG): *Euclea natalensis* extract gel, pH 4.1; (CG): control gel, pH 4.1. The gels were applied to the occlusal slide of the dentin under the following conditions: after 37% phosphoric acid and before 6% citric acid. The hydraulic conductance (HC) of each condition was determined four times using a fluid flow apparatus (Flodec). The data were analyzed using Two-way ANOVA and Tukey's test (*P* < 0.05). *Results*. The greatest mean reduction in HC was produced in group EG dentin discs (61.2%; *P* < 0.05). Even after acid challenge with 6% citric acid the great reduction occurred in group EG (66.0%; *P* < 0.05) than other groups (CG-77.1%, FG-90.8%). *Conclusion*. *E. natalensis* gel not only reduced dentin permeability, but also resisted posttreatment citric acid challenge without changing its permeability. Further research has to confirm this promising result in the clinical situation.

## 1. Introduction

Dentin hypersensitivity is a painful clinical condition, which affects between 4 and 5% of the adult population and is associated with dentin exposure to the oral environment [1–3]. The hydrodynamic theory predicts that exposure of dentin surfaces as a result of enamel loss and/or gingival root surface exposure resulting from attrition, abrasion, erosion, abfraction, or gingival recession can cause sensitivity [3, 4]. Thus, the concept of tubule occlusion as method of dentin desensitization is a logical correlation to the hydrodynamic theory [5]. The fact that many of the agents clinically used to desensitize dentine are effective in reducing dentin permeability tends to support the hydrodynamic theory [6]. Many agents and therapies have been proposed for the treatment of hypersensitivity, however none of them has been proven completely efficacious for such use [7], and new desensitizing agents need to be developed.

In the field of oral health researches, investigations about the contribution of natural products to the treatment of different oral diseases, such as propolis [8] and neem [9], have used experimental formulations and found that they did not cause significant side effects.

*Euclea natalensis* is a plant species that belongs to the family *Ebenaceae* common in tropical and subtropical regions of Africa, specifically on the east coast of Africa, popularly known as *Mulala* [10], Africans have shown the antimicrobial potential of *E. natalensis* roots used for oral care once daily in the morning, soon after breakfast.

A study conducted by Homer et al. [11] demonstrated that the twigs of the plant *E. natalensis* have sufficient antibacterial inhibitory action to interfere in virulence and growth periodontopathic bacteria, *in vivo*. 

 Several studies have evaluated the components present in the *E. natalensis* plant, which may be able to reduce dentin hypersensitivity. Scientific evidences have shown that *E. natalensis* has cytostatic properties [12], low toxicity in healthy tissues, and anti-inflammatory action [13]. 

Considering that the *E. natalenis* is used in different African provinces, and no data have yet been found on the subject in the scientific literature, it would be important to analyze the possibility of using *E. natalensis* for the prevention and/or control of noncarious lesions and dentin hypersensitivity. Thus, the aim of this study was to evaluate the variations in hydraulic conductance of dentin after treatment with *E. natalensis* gel and acidified fluorophosphate gel, *in vitro*. The null hypothesis tested was that the *E. natalensis* gel would not reduce the hydraulic conductance of dentin, *in vitro*.

## 2. Methods

### 2.1. Specimen Preparation and Application of Desensitizing Agents

This research was approved by the Local Research Ethics Committee (Protocol no. 178/2009). The teeth were obtained from the Human Tooth Bank of Dentistry School.

 Freshly extracted human teeth are a potential source of biological pathogens [14]. Extracted human third molars were stored at 4°C in 0.1% thymol (Merck KGaA, Frankfurter Str, Darmstadt, Germany) to inhibit microbial growth and were used within 30 days after extraction.

The crowns were sectioned with a diamond saw in a precision cutting machine (Isomet 1000; Buehler, Lake Bluff, IL, USA) perpendicular to the long axis of the roots to create dentin discs from midcoronal dentin. Thirty-six dentin discs were obtained from the extracted teeth and 30 were used. The smear layer created by the diamond saw was removed with 400–600 grit SiC abrasive paper (Buehler), resulting in dentin discs approximately 0.98 ± 0.08 mm thick, as measured with a micrometer accurate to 0.01 mm. Disc surface was free of coronal enamel and with no evidence of pulp horns [7]. The specimens were immersed in 37% phosphoric acid solution for 15 s to remove the 600-grit SiC smear layer on both sides of the discs. Using 320-grit SiC abrasive paper in a rotary polisher (125 rpm) for 5 s, a standard smear layer was then produced on the occlusal surface of the discs. 

To sample calculate was adopted a *α* error of 5% and a *β* error of 20%, and assumed an estimated six disks per group (SD ± 1.1).

### 2.2. Permeability Measurements

The rate of fluid flow through a dentin specimen was measured using the Flodec device (DeMarco Engineering, Geneva, Switzerland), which follows the movement of a tiny air bubble as it passes down a 0.6 mm diameter glass capillary located between a deionized water reservoir under 140 cm (2 psi) of water pressure and the dentin specimens [15, 16]. An infrared light source passes through the capillary and is detected by a diode, allowing the unit to follow the progress of the air bubble along the length of the capillary. Linear displacement is automatically converted to volume displacement per unit time, from which the instantaneous volumetric flow rate is calculated and logged into a spreadsheet. Flow was measured until a steady-state was reached, typically 0–5 min; then the flow was measured for at least 3 min. Since one datum was taken every second, this resulted in at least 100 readings for each condition (Figure 1). Permeability was expressed as a fluid flow rate in *μ*L min^−1^. All teeth were acid-etched with 37% phosphoric acid for 30 s to ensure maximum permeability was achieved for each specimen. After etching, dentin permeability was determined. The permeability of smear layer etched dentin established a minimum permeability value for that specimen. The permeability of acid-etched dentin established the maximum permeability of each specimens [17].

### 2.3. Application of Materials

The 30 dentin discs were randomly divided into 3 groups of 10 specimens each, corresponding to experimental group (EG): *Euclea natalenis* gel, group F (FG): Fluoride gel 1.23% and group C (CG): treatment with control gel. The materials used were acidulated fluorophosphate gel (1.23% acidulated fluorophosphate, pH 4.1), *E. natalensis* gel (10% of alcoholic extract of *E. natalensis*, pH 4.1), and control gel (base compounds, pH 4.1) (Table 1). The 1.23% fluoride gel was used as a control group as in other studies [7, 18] on treatment for dentin hypersensitivity.

*E. natalensis* was kindly provided by Oral Health Department of Health Ministry of Mozambique and plant identified by Laboratory of Natural Products at Federal University of São Carlos.

The gel of *E. natalensis* was prepared from the dried roots of *E. natalensis* (under controlled parameters) and the *E. natalensis* extract was prepared by macerating 20.0 g of dry powder of *E. natalensis* root with 100 mL of 70% (w/v) ethyl alcohol for a week in a round bottom flask with occasional shaking. The flask was kept under dark to avoid effect of light on the active ingredients of the *E. natalensis*. The extract was then filtered through a muslin cloth for coarse residue and finally through Whatman no. 1 filter paper, measured and kept in an airtight amber colored container. Gel formulation included 10% *E. natalensis* extract, Carbopol, methylparaben, EDTA and sodium hydroxide solution. 

All the desensitizing agents were applied for 4 min, following the manufacturer's instructions for fluorophosphate-gel and then rinsed with deionized water. After the hydraulic conductance was measured under the above conditions, the specimens were exposed to 6% citric acid pH 2.1 for 1 min and the hydraulic conductance was measured again. The aim of this treatment was to evaluate the resistance of the possible occlusive effect of the studied materials to an acidic environment, similar to that found in the mouth. The hydraulic conductance of each condition was determined four times in succession and then the mean value of the maximum Lp was calculated. 

### 2.4. Statistical Analysis

The hydraulic conductivity measurement was performed immediately after treatment application, calculated in mL/min, and expressed as a percentage of maximum permeability obtained after etching. For each specimen, the permeability was measured four times: (1) afterthe smear layer creation, (2) after acid etching of dentin, (3) after applying the gel, and (4) after conditioning with citric acid.

Statistica 9.1 software (Stat Soft, USA) was used. The data were tested by two-way Analysis of Variance (ANOVA), at a 5% level of significance, applied to the reductions in hydraulic conductance, in order to detect differences between the conditions studied. Significant differences were found between materials, conditions, and interaction materials X conditions. Differences were identified by individual comparisons using Tukey's test at a 5% level of significance.

## 3. Results

The effectiveness of the three gels in reducing dentin permeability was analyzed by performing ANOVA for two criteria (*P* < 0.05) (Table 2). Significant differences in the reduction of dentin permeability were found among the tested gels and conditions (*P* < 0.000).

The results showed that although the procedures caused some reduction in the hydraulic conductance of dentin etched with phosphoric acid, the groups presented significant reduction when compared with each other (*P* < 0.05). Tukey's analysis identified significant differences between interactions (conditions and gels) (*P* < 0.05). 

Table 3 shows the mean hydraulic conductance (±SD) of the groups. The desensitizing effects of gels were observed for the groups (CG = 1.63 ± 1.18; FG = 6.29 ± 2.94; EG = 0.92 ± 0.69), which behaved differently and differed significantly from each other. 

There was significant difference in dentin permeability between smear layer and tested gels (*P* < 0.05). Table 3 shows that the effect of gels after citric acid challenge revealed differences among the groups (CG = 77.1%; FG = 90.8%; EG = 66.0%) (*P* < 0.05). The EG group provided a reduction in permeability even after the acid challenge.

## 4. Discussion

There are diverse indications for the use of plant extracts, with very common multiplant regimens used in many traditional South African medicinal treatments. Several African tribes use the common traditional chewing stick scientifically known as *E. natalensis* [19]. The present plant extracts showed moderate cytotoxicity on the Vero cell line [20]. 

Natural products, such as propolis gel [8], have been developed to reduce dentin hypersensitivity. Nevertheless, therapeutic intervention with desensitizing agents may provide only partial pain relief and recurrence is common [21, 22]. 

In the present study, gel was used as a vehicle to deliver *E. natalensis* to the dental structure, in order to prevent further dentin permeability. Thus the null hypothesis was rejected.

The FG and EG presented significant difference from CG (*P* < 0.05) in the reduction of dentin permeability. Treatment in the control group was based on gel, prepared with same compounds as used for the FG and EG, but without the therapeutic agents. The physical benefit provided by the vehicle was similar in all the groups, removing the intergroup error analysis. The fluoride gel was worse for preventing dentin permeability (90.8%), followed by the control gel (77.1%), and the *E. natalensis* was the most effective (66.0%). Among the conditions, there was no significant difference as regards smear layer, gels, and acid challenge, except for 37% phosphoric acid (*P* < 0.05). 

*E. natalensis* presented the most effective action to reduce dentin permeability. This effect can be attributed to the flavonoids, taninus, and naphthoquinones present in the plant roots [10]. These *E. natalensis* compounds may be responsible for the dentin tubule obliteration due to the formation of a protective layer on the teeth [23]. 

A survey of the literature has shown that natural products such as flavonoids [24], terpenoids, naphthoquinones acetylenes, and tropolones have been identified. Naphthoquinones are widely distributed in plants [25] and many are found to exhibit an interesting range of pharmacological properties including antibacterial [26], antiviral [27], trypanocidal [28], anticancer [29], and antifungal activity [30, 31].

Naphthoquinone 7-methyljuglone (5-hydroxy-7-methyl-1,4-aphthoquinone) has previously been isolated and identified as an active component of root extracts of *E. natalensis* [32], which could be considered the most active compound [10]. This compound may act as a potent antioxidant which significantly interferes with the apoptotic event [33]. 

The use of citric acid after the experimental gels is made in order to simulate the gel strength of the acid attacks normally undergoes a tooth when present in the oral cavity during ingestion of food or beverages. The results showed no significant difference between the values obtained after the application of gels and after application of citric acid, which proves that all the gels tested offered some resistance to acid challenge. The protection of the *E. natalensis* gel may be due to presence of tannins and flavonoids. Tannins supposedly have an astringent effect on the mucous membrane [34, 35], and the interaction of tannins with salivary proteins causes the aggregation and precipitation of protein-tannin complexes [35] that form a layer over enamel, thus providing protection against dental caries [36], and this property could also help to prevent dental wear [23, 37]. The organic degradation of dentin might also be affected by other host-derived enzymes, such as matrix metalloproteinases (MMPs), which are present in saliva and dental hard tissues [38]. Some flavonoids, as green tea polyphenols, could inhibit activity against MMPs [37, 38]. 

The limitations imposed by the method should be considered, thus they depended on an initial clustering of the specimens, which were standardized for all other comparisons, starting with the smear layer, phosphoric acid gel and finally citric acid application [39]. *In vitro* method is an initial phase to test a new product to a problem, thus many characteristics of *in vivo* methods, as the presence of saliva, is difficult to be reproduced in the laboratory. Thus others studies, such in situ, should be developed to get results more compatible to clinical environment. 

The minimum permeability of the specimens is determined by the presence of the smear layer occluding the dentin tubules, allowing minimal movement of fluids through the dentin. One study reported that the presence of smear layer on the surface of dentin is responsible for most of the total resistance to the movement of fluids within the dentin. The maximum permeability is determined by removing the smear layer by demineralization, which causes a significant increase in the filtration of fluid through the dentin [40]. 

*E. natalensis* causes light yellow-spots on the teeth and in the mouth. This transitory staining [13] is caused by flavonoids, however, it disappear within hours [20]. The colors of flavonoids are directly related to the environment and show an intense yellow at an alkaline pH and disappear in the presence of acid [41]. 

*E. natalensis* gel exhibited good activity after acid challenge to reduce dentin permeability, while maintaining similar protection when applying the gel. Further studies *in vitro* and *in situ* are needed to evaluate the properties of the *E. natalensis* extract effect on dentin permeability. This present research has pioneered the use of gel containing *E. natalensis* as a treatment for dentin hypersensitivity. 

 These findings are very important, especially for public health in Africa, where the *E. natalensis* roots are easily obtainable and used as tools for performing oral hygiene. There are additional benefits, as the *E. natalensis* root extract is a natural remedy for diarrhea, gonorrhea, bronchitis, pleurisy, asthma, chronic urinary tract infections, and for relieving headache and toothache [42], and also contributes to oral health.

## 5. Conclusion

Within the limitations of this study, the experimental *E. natalensis* gel formulation can interfere in the reduction/prevention of dentin permeability, even when submitted to acids challenges, and therefore the null hypothesis tested was rejected. The* E. natalensis* gel has provided a mechanical blocking of the experimental dentin specimen. Plant extracts used traditionally for the prevention and treatment of oral problems could be used to reduce dentin hypersensitivity. Further research has to confirm this promising result in the clinical situation.

## Figures and Tables

**Figure 1:** Permeability measurements adapted of Rusin et al. [15].

**Table 1:** Experimental design.

Treatments	Dentinal permeability (Lp) evaluations
Smear layer (400 grit, wet sanding for 30 s)	Minimum Lp
37% phosphoric acid (application for 30 s)	Maximum Lp (Lp 100%)
Product (application for 4 min)	Lp reduction
Citric acid solution 0.02 M pH 2.5 at 37-38°C (exposure for 1 min)	Lp variation

Lp: Hydraulic conductance.

**Table 2:** The gels were compared to the reductions in dentinal permeability between the conditions by two-way ANOVA.

	df	MS	df	SS	*F*-ratio	*P*
	effect	effect	error	error		
Gels	2	187.9275	36	3.0799	49.1870	0.0000*
Conditions	3	63.6139	116	10.0409	16.6481	0.00000*
Interaction	6	18.5951	108	4.9125	4.8664	0.00011*

df: Degrees of freedom; MS: Mean square; SS: Standard error.

*Significant differences.

**Table 3:** Means (%) of hydraulic conductance (±SD) for each gels type as an after acid challenge as well as minimum and maximum (100%) hydraulic conductance and Tukey's test compared.

		Hydraulic conductance	
Groups	Conditions	values %	*μ*L min^−1^ 140 cm H_2_O^−1^
Control group (base gel)	Smear layer-covered dentin	100.0	2.47 ± 1.32^A^
	37% PA etched dentin	9.2	0.20 ± 0.22^B^
	Treatment with control gel	73.8	1.63 ± 1.18^Aa^
	Posttreatment 6% CA etched	1.90	1.90 ± 0.51^A^

Fluoride gel group	Smear layer-covered dentin	100.0	7.04 ± 1.53^C^
	37% PA etched dentin	10.5	0.60 ± 0.83^B^
	Treatment with F gel	89.3	6.29 ± 1.94^Cb^
	Posttreatment 6% CA etched	90.8	6.32 ± 1.77^C^

*Euclea natalensis* gel group	Smear layer-covered dentin	100.0	2.53 ± 1.15^A^
	37% PA etched dentin	20.1	0.36 ± 0.50^B^
	Treatment with EN gel	61.2	0.92 ± 0.69^Bc^
	Posttreatment 6% CA etched	66.0	1.01 ± 0.70^B^

*Different lower case letters in the same column indicate statistical significance between the gels. Different upper case letters in the same column indicate statistical significance among the different conditions (*P* < 0.05).
